This article has been retracted.

# Scanning Imaging Study of Patients with Parkinson's Disease Lower Urinary Tract Dysfunction Based on Linear Equation

**DOI:** 10.1155/2022/9506328

**Published:** 2022-05-27

**Authors:** Yong Liu, Jiasheng Han, Xuguang Guo, Lei Fang, Ting Liu

**Affiliations:** ^1^Neurology Department, The 80th Group Army Hospital of the People's Liberation Army, Weifang, Shandong 261021, China; ^2^Urinary Surgery, The 80th Group Army Hospital of the People's Liberation Army, Weifang, Shandong 261021, China; ^3^School of Public Health, Weifang Medical College, Weifang, Shandong 261021, China

## Abstract

A predictive method based on a linear equation was proposed to study the factors influencing lower urinary tract dysfunction in Parkinson's disease. A 10-month follow-up of 200 selected Parkinson's patients from January to December 2020 used a linear regression equation to analyze whether depletion function was associated with a specific nonmotor function loss, and a linear regression equation was used for analysis. A loss of emptiness function was used to determine whether there are complications associated with lower motor function and cognitive function. The experimental results showed that dysuria in Parkinson's disease was related to the following nonmotility disorders: gastrointestinal dysfunction (OR 2.52, 95% CI 1.57-3.92, *P* < 0.001), cardiovascular dysfunction (OR 2.31, 95% CI 1.23~4.11, *P* = 0.014), respiratory dysfunction (OR 1.72, 95% CI 1.32~3.24, *P* = 0.029), cutaneous autonomic dysfunction (OR 1.91, 95% CI 1.15~3.08, *P* = 0.023), and sleep disorders (OR 2.01, 95% CI 1.32~3.14, *P* = 0.001). In addition, dysuria was associated with higher UPDRS-III (regression coefficient 1.74, 95% CI 0.56-2.67, *P* = 0.001). Thus, nonmotor disorders have been shown to be associated with early impairment.

## 1. Introduction

Parkinson's disease (PD) is a progressive degenerative disease of the central nervous system; its typical symptom is motor dysfunction, which mainly includes motor retardation, muscle rigidity, resting tremor, and ataxia. For a long time, the treatment of PD is mainly to improve motor symptoms [1]. A large-scale epidemiological survey showed that, for 206 cases in 2019, 304 cases in 2018, and 404 cases in 2017, the incidence of lower urinary tract dysfunction in PD patients is as high as 27.0% to 63.9%, mainly including overactive bladder (OAB), nocturia, urge incontinence (UI), and detrusor overactivity [2]. In addition, some patients will have slight urinary tract obstruction. Lower urinary tract function involves the regulation of multiple nerve pathways, and the mechanism of lower urinary tract dysfunction in PD patients is complicated; the current study believes that it may be due to basal ganglia disease in PD patients, interfering with the function of the pontine voiding center. Studies have shown that about 90% of Parkinson's patients will have some degree of speech disorder; therefore, it is more convenient and effective to directly collect voices for research through noncontact methods, such as array microphones, compared with other diagnostic methods. This has caused great attention on the research on voice-based Parkinson's diagnosis and treatment programs. With the rapid development of computer technology, in recent years, people have applied many diagnosis and treatment programs based on machine learning algorithms to study Parkinson's disease, in order to completely replace clinical decision-making [3]. These diagnosis and treatment plans are mainly classified into two categories: (1) determining whether the user has Parkinson's disease, that is, realizing the diagnosis of Parkinson's disease (the common one is based on the linearly separable and nonlinear separable data and linear SVM and nonlinear SVM application for research); (2) predicting the severity of Parkinson's disease patients, that is, tracking the progress of Parkinson's disease by predicting UPDRS (unified Parkinson's disease rating scale) [4].

24-month follow-up data showed that the prevalence of early urinary dysfunction in Parkinson's is stable at about 50%. In the study, the lowest rate of patients with urination disorders was 47.86% (T1) and the highest was 51.28% (T2); it is basically consistent with the research results of Picillo et al. The above data shows that urination disorders can appear in the early stage of the disease and basically remained stable as the disease progressed; it further supports that Parkinson's disease dysuria may be related to early autonomic nerve damage [5]. However, Senol's statistical study showed that Parkinson's patients with urinary dysfunction accounted for 63.9%. The reason for the difference in the above data may be that Picillo et al. and this study are both the results of the statistics of Parkinson's early urinary dysfunction; the entire natural history of the development and evolution of urination disorders is not covered [6]. Research by Lindsay et al. showed that patients with Parkinson's urinary dysfunction had more nonmotor symptoms than those without urinary dysfunction [7]. Based on this, the study conducted a 10-month follow-up observation of 200 Parkinson's disease patients selected from January to December 2020; linear regression equation was used to analyze whether urinary dysfunction is related to specific nonmotor dysfunction and to analyze whether urinary dysfunction is related to lower motor function and cognitive function. Prospective data analysis was used in order to clarify the marker role of Parkinson's early urination disorder in the progression of dysfunction (nondyskinesia and dyskinesia).

## 2. Prediction of Parkinson's Disease UPDRS Based on GBDT

### 2.1. Data Set Description

This article uses the remote Parkinson's data set in UCI, which contains 42 speech samples with Parkinson's disease; the sample is derived from the continuous vowel/a/voice collected from the patient once a week, collected 6 pieces each time, lasting 6 months, at a total of 5875 samples. Through the speech signal processing algorithm, the total number of features extracted from these speech samples is 16; among them, the characteristics that measure the change of the fundamental frequency are as follows: jitter (%), jitter absolute value (Abs), relative amplitude perturbation jitter (RAP), 5-point period perturbation entropy jitter (PPQ5), and absolute difference of the period and the average period ratio jitter (DDP); the characteristics that measure the amplitude change are as follows: local flicker (dB) shimmer (dB), 3-point amplitude perturbation entropy shimmer (APQ3), 5-point amplitude perturbation entropy shimmer (APQ5), 11-point amplitude perturbation entropy shimmer (APQ11), average absolute difference of the amplitude difference between adjacent period shimmer (DDA), noise harmonic ratio (NHR), harmonic noise ratio (HNR), cyclic period density entropy (RPDE), trend fluctuation analysis (DFA), and pitch period entropy (PPE). And finally, a sample set of5875∗16is obtained [8].

### 2.2. Data Set Division

Computers can use machine learning to construct various linear regression equations to solve the same or similar problems. However, for the establishment of a good linear regression equation, in addition to relying on a suitable algorithm, the computing power of the computer also requires data preprocessing for the data set. Using the remote Parkinson data set in UCI and using LS to train the prediction model, a certain prediction effect has been achieved. In this article, two different data sets are taken as examples, using ordinary least squares to train a regression prediction model, model 3, as shown in Figure 1. Taking into account the distribution of sample data, obviously, model 3 has made a compromise in order to fit object samples in two different domains; the real prediction effect of this model is not very satisfactory. The learning of the regression model is to calculate the square error between the predicted value and the true value of all data, and the error is accumulated so that the positive difference and the negative difference cancel each other out. This will lead to regression prediction on sample data sets with different distributions, that is, different domains, but the same model can be obtained. The concept of data set distribution is more complicated; in general, the sample size of each type should be conducive to the establishment and evaluation of the model [9]. According to the principle of Occam's razor, when choosing a model, a very simple model that can interpret the known data well is the most suitable model [10]. Analyzing the remote Parkinson data set, the model 3 built on these two objects is obviously underfitting, but if the two objects are divided into two domains of data according to a certain prior knowledge and then the original model is decomposed on the two domains, then the model 1 and model 2 established on the two domains can fit the data in the respective domains well, as shown in Figure 1. Therefore, the data set is divided according to the gender and age of the object, and linear regression equations are established on different data sets to achieve effective decomposition [11]. In practical applications, the user's voice is collected, and according to the user's age and gender, a suitable model is given through the recommendation system to realize the prediction of the user's UPDRS. The principle is shown in Figure 2.

### 2.3. Iterative Decision Tree

Integrated learning can significantly improve the generalization ability of the learning system; it has received extensive attention from the linear regression equation community. GBDT is an integrated learning algorithm; a strong learner is generated by the combination of multiple weak learners. The algorithm is continuously iterated by multiple decision trees; through iteration, the linear regression and residuals of all trees are equal to or approaching 0, and a high-accuracy prediction model is finally obtained.

Assume that the initially obtained learner is

(1) $$\begin{array}{c} F_{0}\left(x\right)=agr\underset{a}{\min}\overset{n}{\underset{i=1}{\sum }}L\left(y_{i},a\right). \end{array}$$

Among them, *L*(*y*_*i*_, *a*) is the loss function of model *f*(*x*). ((*x*_*i*_, *y*_*i*_))_*i*=1_^*n*^ is the sample training set, *x*_*i*_ is the feature, and the corresponding result is *y*_*i*_.

First, according to the current data, the loss function is minimized, and the initial loss function model is obtained. The number of iterations is set to *M*; each iteration produces a model, in order to minimize the loss function of the model generated in each iteration to the training set, according to equation (1); in each iteration, the loss function is made smaller and smaller by moving to the negative gradient direction of the loss function, to get more and more accurate models. The main steps of algorithm iteration are as follows.

The first step is to calculate the residual *r*_*a*_.

Use the initial model *F*_0_(*x*) to calculate the negative gradient, as shown in equation (2). The negative gradient of the loss function is used as the residual for the current model *F*_0_(*x*) value. For the square loss function, this value is the residual, and for the general loss function, this value is the estimated value of the residual.

(2) $$\begin{array}{c} r_{i1}=-\left[\frac{\partial L\left(y_{i},F_{0}\left(x_{i}\right)\right)}{\partial F_{0}\left(x_{i}\right)}\right],\;i=1,2,\cdots ,n. \end{array}$$

The second step is to train a linear regression equation and get the decision tree *h*_1_(*x*) composed of leaf nodes.

The third step is to find a suitable step length. In the gradient descent used in the GBDT algorithm, the step size is obtained by calculation. The calculation rule is to minimize the *F*_1_(*x*) loss function *β*_1_ value of the new learner.

(3) $$\begin{array}{c} \beta_{1}=agr\underset{a}{\min}\overset{n}{\underset{i=1}{\sum }}L\left(y_{i},F_{0}\left(x_{i}\right)+{ah}_{1}\left(x_{i}\right)\right). \end{array}$$

The fourth step, according to the gradient and step length, is to iteratively obtain the regression tree model *F*_1_(*x*), as shown in the following equation:

(4) $$\begin{array}{c} F_{1}\left(x\right)=F_{0}\left(x\right)+\beta_{1}h_{1}\left(x\right). \end{array}$$

Through the above four steps, the second model *F*_1_(*x*) can be optimized from the initial model *F*_0_(*x*). Iterate these four steps *M* − 1 times to get the final GBDT model.

## 3. Experimental Analysis

### 3.1. Data Preprocessing

Data preprocessing generally includes operations such as feature selection and data cleaning. Feature selection refers to selecting a subset of important features from the original feature set. Feature selection can remove redundant or irrelevant features, in order to achieve the purpose of improving the generalization ability of the model. The feature selection algorithm used in this article is Relief [12]. The earliest Relief algorithm was used to solve the problem of two classifications, the algorithm designs a relevant statistical vector to evaluate the importance of each feature, each component of the vector is the evaluation value of one of the initial features, the importance of a feature subset is the sum of relevant statistics of all features in the subset, and this correlation statistic is regarded as the weight of each feature; that is, Relief belongs to a feature weighting algorithm. The formula is as follows:

(5) $$\begin{array}{c} W\left(f_{j}\right)=\frac{1}{q}\overset{q}{\underset{i=1}{\sum }}\left\{-\frac{1}{\left|NH\left(X_{i}\right)\right|}\cdot \underset{X_{n}\in NH\left(X_{i}\right)}{\sum }\left\|x_{i,j}-x_{n,j}\right\|+\underset{y_{l}\neq y_{i}}{\sum }\frac{1}{\left|NM\left(X_{i}\right)\right|}\cdot \frac{p\left(y=y_{l}\right)}{1-p\left(y=y_{l}\right)}\cdot \underset{X_{n}\in NH\left(X_{i}\right)}{\sum }\left\|x_{i,j}-x_{n,j}\right\|\right\}. \end{array}$$

Among them, *W*(*f*_*j*_) represents the weight of the *j*-th feature, *q* represents the number of samples randomly selected, *X*_*i*_ represents a data sample, |*NH*(*X*_*i*_)| represents the number of similar samples closest to sample *X*_*i*_, |*NH*(*X*_*i*_)| represents the number of different types of samples closest to the sample *X*_*i*_, and ‖·‖ represents the distance measurement, commonly using the Euclidean distance or Manhattan distance. Use the Relief algorithm to get feature weights; the importance of the features is sorted according to the weight, and the top 13 important features are selected. After the feature selection is completed, the data cannot be directly used for calculation; in many cases, some basic processing of the data is required [13]. These basic processing includes the processing of missing values, the processing of nondigital feature values, and the processing of outliers; the remote Parkinson data set has been cleaned up.

### 3.2. Statistical Methods

Perform a normal distribution test on the collected data; subsequently, the data of PD-UD and PD-NUD groups were subjected to *χ*^2^ test, *t* test, and one-way analysis of variance (ANOVA) according to the situation. The results are expressed in percentage (%), mean, and standard deviation (SD) (*x* ± *s*). To examine the relationship between nonmotor dysfunction and early urination disorders, multivariate mixed-effect linear regression equations were used to control independent variables such as age and UPDRS-III. To examine the relationship between motor function, cognitive function, and early voiding dysfunction, multiple mixed-effect linear regression analysis was performed, with gender and age as covariates, and covariance analysis was performed. All covariates were tested for multicollinearity. When the variance inflation factor is less than 5, all predictors can be considered independent. The analysis result is expressed by odds ratio (OR) and regression coefficient. The study used 95% confidence interval (CI); *P* ≤ 0.05 as the difference was statistically significant [14].

### 3.3. Experimental Method

Each patient undergoes 3 data collections: T1 (baseline value), T2 (3 months), and T3 (9 months). During the follow-up period, if the patient develops other diseases (such as cerebral infarction, cerebral hemorrhage, and cerebellar atrophy) that may affect motor, nonmotor functions, and urinary symptoms, and if it is difficult to distinguish symptoms that affects the accuracy of the data, the sample will be eliminated. Each data collection includes the following:

1. Collect samples for urination disorders. Those who have one of the following symptoms and last for more than 3 months can be considered as combined urination disorders: (1) urgency, (2) frequent urination (≥1 time/2 h), and (3) nocturia. Patients with positive results were classified into the urinary dysfunction group (PD-UD), and the rest were classified into the nonurinary dysfunction group (PD-NUD).
2. Investigate the following 6 nonmotor dysfunctions through face-to-face interviews: gastrointestinal dysfunction, cardiovascular dysfunction, sleep disorders, respiratory dysfunction, mental disorders, and skin lesions. Each NMS includes several specific questions, and the answers are all divided into two parts (“yes” or “no”).
3. The motor function level of the samples was evaluated by the unified Parkinson's disease rating scale 3.0 (UPDRS-III). The higher the UPDRS-III score, the lower the patient's motor function level

## 4. Experimental Results

A total of 204 of 324 Parkinson's patients passed the screening. During the 9-month observation period, 4 cases were excluded due to new cerebral infarction, and the final sample count was 200 cases [15]. During the entire observation period, the lowest prevalence of urination disorders was T147.86%, and the highest was T251.28%. Data are shown 3 times, the PD-UD group is usually older and more male, and the UPDRS-III score is higher than that of the PD-NUD group. The prevalence of almost all nonmovement disorders in the PD-UD group was higher than that in the PD-NUD group, and the difference was statistically significant (*P* < 0.05) [16]. After linear regression analysis, the following nonmotility disorders may be associated with early voiding disorders: gastrointestinal dysfunction (OR 2.52, 95% CI 1.57-3.92, *P* < 0.001), cardiovascular dysfunction (OR 2.31, 95% CI 1.23-4.11, *P* = 0.014), sleep disturbance (OR 2.01, 95% CI 1.32~3.14, *P* = 0.001), respiratory dysfunction (OR 1.72, 95% CI 1.32~3.24, *P* = 0.029), and autonomous skin disease (OR 1.91, 95% CI 1.15-3.08, *P* = 0.023).  Figure 3 shows a comparison of the degree of motor function between PD-NUD and PD-UD during the observation period. In the three sets of data, both T1 and T2 showed that there was no statistical difference in the relationship between mental disorders and urinary system diseases. Multiple linear regression analysis showed that compared with PD-NUD, early voiding disturbance was associated with higher UPDRS-III (regression coefficient 1.74, 95% CI 0.56-2.67, *P* = 0.001) [17].

Figure 4 Comparison of the cognitive function of PD-NUD and PD-UD during the observation period, It can be clearly seen from Figure 3 that the reduction in motor function level in the PD-UD group was more significant within 9 months. A recent domestic study shows that the untreated Parkinson's overactive bladder symptom score (OABSS score) was positively correlated with the UP-DRS-III score and the hypoactive rigidity score. The study also showed that the degree of dyskinesia and the use of levodopa in Parkinson's patients with urinary dysfunction increased significantly after 24 months. Consistent with the above conclusions, the study also confirmed the link between early urination disorders and lower levels of motor function [18]. The study also showed that early urination disorders are related to the following nondyskinesias through linear regression equation analysis, including gastrointestinal dysfunction (OR 2.52, 95% CI 1.57~3.92, *P* < 0.001), cardiovascular dysfunction (OR 2.31, 95% CI 1.23~4.11, *P* = 0.014), respiratory dysfunction (OR 1.72, 95% CI 1.32~3.24, *P* = 0.029), autonomic skin disorders (OR 1.91, 95% CI 1.15~3.08, *P* = 0.023), and sleep disturbance (OR 2.01, 95% CI 1.32~3.14, *P* = 0.001). Among them, gastrointestinal dysfunction, cardiovascular dysfunction, skin lesions, and urination disorders are all autonomic nerve dysfunction. Studies have shown that the cause of urinary disturbance and sleep disturbance may be related to brainstem lesions in the early stage of the disease [19]. As can be seen from Figure 4, the score of the PD-UD group decreased more significantly than that of the PD-NUD group within 9 months, and linear regression analysis also showed dysuria (regression coefficient -0.21, 95% CI -0.87~0.22, *P* = 0.043), the research conclusions were inconsistent (regression coefficient -0.34, 95% CI -0.92~0.24, *P* = 0.251), and there was no statistical difference between the two. Therefore, the correlation between early Parkinsonian urinary dysfunction and cognitive function level still needs high-level research to continue [20].

## 5. Conclusion

Studies have shown that urinary dysfunction in Parkinson's disease can be used as an early clinical indicator of the progression of dyskinesia and nondyskinesia. Experimental results show that the final prediction effect is more than half that of the ordinary decision tree; at the same time, it has been further verified that Parkinson's disease is greatly affected by age and gender. Gender and age belong to prior knowledge; using these kinds of prior knowledge to decompose prediction models not only is simple and efficient but also has certain practical guiding significance. Of course, in addition to gender, there are many other kinds of a priori knowledge of life, such as the patient's health status, loss of gastrointestinal function, cardiovascular dysfunction, skin lesions, and sleep disorders. Many of these are associated with loss of autonomic function, which to some extent supports the classification of nonmotor symptoms of Parkinson's disease. The functional classification is long. Sufficient classification of Parkinson's disease, in particular, a comprehensive assessment system covering motor and nonmotor functions, is needed.

## Figures and Tables

**Figure 1:** Regression training model.

**Figure 2:** Implementation process.

**Figure 3:** Comparison of the degree of motor function between PD-NUD and PD-UD during the observation period.

**Figure 4:** Comparison of the cognitive function of PD-NUD and PD-UD during the observation period.

## Data Availability

The data used to support the findings of this study are available from the corresponding author upon request.
